The article "Serosurvey of Cystic Echinococcosis and Related Risk Factors for Infection in Fars Province, Southern Iran: A Population-Based Study" was published in 2022. Journal: Biomed Res Int.

# Serosurvey of Cystic Echinococcosis and Related Risk Factors for Infection in Fars Province, Southern Iran: A Population-Based Study

**DOI:** 10.1155/2022/3709694

**Published:** 2022-09-05

**Authors:** Ali Reza Safarpour, Mostafa Omidian, Ali Pouryousef, Mohammad Reza Fattahi, Bahador Sarkari

**Affiliations:** ^1^Gastroenterology Research Center, Shiraz University of Medical Sciences, Shiraz, Iran; ^2^Department of Parasitology and Mycology, School of Medicine, Shiraz University of Medical Sciences, Shiraz, Iran

## Abstract

Cystic echinococcosis (CE) is a common zoonotic infection in all provinces of Iran, especially in areas where people live on agriculture and animal husbandry. The current cross-sectional population-based study is aimed at determining the seroprevalence of CE in Kavar County, Fars province, southern Iran. Blood samples were collected from 1500 individuals (749 males and 751 females). Anti-hydatid cyst antibodies were detected, using a recombinant B8/1 antigen of *Echinococcus graunlosus* in an ELISA system. Multivariate logistic regression analysis was used to find out the independent risk factor for CE seropositivity. Anti-hydatid cyst antibodies were detected in the sera of 131 out of 1500 participants, corresponding to a seroprevalence rate of 8.73%. With a statistically significant difference (*p* < 0.05), the seroprevalence of hydatid cyst in males and females was 5% and 7%, respectively. Differences in the seropositivity of hydatid cysts were also statistically significant by occupation (*p* < 0.05). The seroprevalence of hydatid cyst was significantly higher in the age group of 35-45 years than in other age groups (*p* < 0.05). Multivariate logistic regression showed that only age was associated with seropositivity to CE (OR = 2.23, 95% CI: 1.33-3.72). Moreover, there was a statistically significant association between seropositivity to hydatid cysts and underlying diseases such as hypertension (*p* = 0.049) and fatty liver (*p* = 0.048). The findings of this study indicate that the seroprevalence rate of CE is relatively high in the Fars province, southern Iran, and this high rate of infection is mainly linked to people's jobs and lifestyles.

## 1. Introduction

Cystic echinococcosis (CE) is a zoonotic neglected parasitic infection of humans and some other mammals caused by the larval stages of the cestode *Echinococcus granulosus*. CE is one of the most important health challenges in Iran, and the disease exists throughout the 31 provinces of the country. The overall seroprevalence of human hydatid cyst in Iran is reported to be 4.2% while the prevalence of *Echinococcus* infection in definitive hosts is reported to be 23.6% [1]. In Iran, the highest prevalence of hydatid cysts in humans, as well as the highest rate of *Echinococcus* infection in the final hosts (mainly dogs), has been reported in the southern regions of the country [1]. In a study by Asadi et al., on 220 municipal workers in Urmia, northwestern Iran, anti-hydatid cyst antibodies were detected in 2.3% of the studied individuals [2]. In two recent studies conducted in Fars province, southern Iran, the seroprevalence of hydatid cyst among children living in a rural area and blood donors was reported to be 6.7 and 5.6%, respectively [3, 4].

In Iran, about one percent of surgeries performed in hospitals are on patients with hydatid cysts [5]. In addition, it has been estimated that the number of people with asymptomatic hydatid cyst in Iran is about 635,232, and the annual cost of the disease (including direct and indirect costs) is $ 232.3 million [5]. Seroepidemiological studies conducted in different parts of Iran have reported the rate of hydatid cyst from 0.1% to 9.5%. For example, in the study of Harandi et al. in rural areas of Kerman province, in southeast Iran, the seroprevalence rate for hydatid cyst was reported to be 7.3% [6].

Fars province is one of the most important centers of hydatid cysts in Iran due to favorable climatic conditions and the people's livelihood of agriculture and animal husbandry. Although there have been various studies on the prevalence of hydatid cyst in different regions of Iran in different population groups, a comprehensive study that shows the status of this disease in a relatively large population in a society with agricultural and animal husbandry livelihood in Iran, especially in Fars province, as one of the main endemic areas for CE, is missing. Hence, the current study is aimed at assessing the seroprevalence of hydatid cyst and related risk factors for infection in residents of Kavar County in Fars province, where the largest and the most comprehensive Persian population cohort on noncommunicable diseases is running.

## 2. Materials and Methods

### 2.1. Study Area

The present cross-sectional population-based study was performed in collaboration with the Kavar Persian population cohort and the Department of Parasitology at Shiraz University of Medical Sciences, Shiraz, Iran, in Kavar County in Fars province. Two main research centers, the Endocrine Research Center and Gastroenterohepatology Research Center, affiliated with Shiraz University of Medical Sciences (SUMS) are implementing the comprehensive Persian cohort study. Kavar has a population of about 71,856 and is located 35 kilometers southeast of Shiraz the capital of Fars province (Figure 1).

Kavar's geographical coordinates are latitude 11°29′N and longitude 42°52′E. The average annual precipitation and temperature in this area are 400 mm and 22°C, respectively. Kavar County has a large number of stray dogs that are in close contact with humans and other animals, including sheep and goats. On the other hand, the majority of people who live in Kavar, due to their employment in agriculture, horticulture, and animal husbandry, are prone to soil-transmitted parasitic infections, especially hydatid cyst and toxocariasis.

### 2.2. Sample Collection

In coordination with the implementers of the Persian cohort project in Kavar County, blood samples were taken from 1500 participants in the cohort project from the residents of the district. As the participants in the cohort study had a specific code, the participants were randomly selected from the numbers assigned to each person.

Ethical approval of the study was obtained from the Ethical Review Committee of Shiraz University of Medical Sciences (ethical approval code: IR.SUMS.REC.1399.960). After signing a written informed consent and filling out a questionnaire containing sociodemographic data and risk factors related to hydatid cyst, a blood sample (5 mL) was taken from each subject. The isolated sera were kept at -20°C until sampling was completed. Frozen sera were transferred to Shiraz University of Medical Sciences (parasitology laboratory) where the samples were tested for anti-hydatid cyst antibodies.

### 2.3. Detection of Anti-hydatid Cyst Antibodies

*E. granulosus* recombinant B8/1 antigen (rEgAgB8/1) was produced in our previous study which had a sensitivity of 93% and specificity of 92% for the diagnosis of human CE [7]. ELISA with the recombinant antigen was performed in flat-bottom 96-well microplates. The microplate was coated (100 *μ*L/well) with a concentration of 5 *μ*g/mL of the recombinant antigen in 0.1 M carbonate/bicarbonate (coating) buffer at 4°C overnight. The next day, after washing the microplate with PBST (phosphate-buffered saline, containing 0.05% Tween 20), wells were blocked with 3% skimmed milk for 2 h at room temperature (RT). Serum samples (1/100 dilution in PBST) were added to each well and incubated for 1 h at RT. Then, the plates were washed as before, and 100 *μ*L of a predetermined dilution (1/4000) of the horseradish peroxidase-conjugated goat anti-human IgG (Sigma, USA) was added to the wells and incubated at RT for an hour. The plate was washed as before and incubated with a substrate solution containing 0.4 mg/mL OPD and 0.3% H_2_O_2_ in 0.1 M citrate buffer (100 *μ*L/well) for 30 min in darkness at RT. The absorbance at 450 nm was measured, using a microplate reader (ELX800, BioTek, USA). In each run, positive and negative control sera were included. Finally, the cutoff point was set at 2SD from the mean of control samples.

### 2.4. Statistical Analyses

SPSS ver. 20 software (SPSS Inc., Chicago, IL, USA) was applied for statistical analyses of the data. The chi-square test was used to determine the association between the seropositivity to hydatid cyst and individuals' demographic characteristics. Multivariate logistic regression analysis was used to find out the independent risk factor for CE seropositivity in the recruited subjects. Also, univariate logistic regression analysis was employed to determine the association between the different risk factors and seropositivity to CE. Statistical significance was considered as a value of *p* < 0.05.

## 3. Results

Of the 1500 recruited subjects, 749 (49.9%) were males, and 751 (50.1%) were females. The mean age of the subjects was 50.04 (±8.3) years, ranging from 35 to 70 years. Most of the subjects (41.1%) belonged to the 46-55-year-old group. Most of the recruited subjects (32%) were illiterate or had elementary (32.9%) education. Anti-hydatid cyst antibodies were detected in the sera of 131 out of 1500 participants, corresponding to a seroprevalence rate of 8.73%. The seroprevalence rate of hydatid cyst in males and females was 6.94% (52/749) and 10.51% (79/751), respectively, and the difference was statistically significant (*p* = 0.02). Also, seropositivity to hydatid cyst had a statistically significant association with people occupation (*p* = 0.008). The rate of seropositivity was significantly higher among the age group of 35-45 years (*p* = 0.01). Univariate analysis showed a significant association between sex, age, and occupation with seropositivity to hydatid cyst. Multivariate logistic regression analysis indicated that only the age group of 35-45 years with OR = 2.23 (95% CI: 1.33-3.72, *p* = 0.002) was associated with seropositivity to hydatid cyst. It is noteworthy that a statistically significant association was found between seropositivity to hydatid cyst and two underlying diseases, including hypertension (*p* = 0.049) and fatty liver (*p* = 0.048), while the association between seropositivity to hydatid cyst and other underlying diseases, including psychiatric disorder, epilepsy, cancers, rheumatic disease, chronic lung disease, renal disease, cardiac disease, and diabetes, was insignificant (*p* > 0.05).  Table 1 shows the demographic features and relative seropositivity to hydatid cyst in 1500 evaluated subjects in Kavar County, Fars Province, southern Iran.

## 4. Discussion

CE is a zoonotic disease with a worldwide distribution, caused by the larval stage of *E. granulosus*, a cestode belonging to the Taeniidae family [8]. The disease is more common in the Mediterranean region, Central Asia, China, Australia, South America, North and East Africa, and the Middle East [3, 4, 9–13].

Iran is one of the hyperendemic regions of the disease where the disease has been reported in all 31 provinces of the country. Despite conducting several studies on the seroprevalence of hydatid cysts in Iran, a comprehensive study has not been conducted on the status of this disease in a relatively large population with a specific agricultural and animal husbandry livelihood. This lack of information justified the current study which assessed the seroprevalence of CE in a relatively large population in Fars province, southern Iran.

The prevalence of anti-hydatid cyst antibodies in the present study among the population of the study area, Kavar County in Fars province, was 8.73%. This rate is in line with the studies conducted in other areas of Iran, including Yasuj (7.2-8.1%) in the Zagros Mountains of southwestern Iran, Khuzestan in the south (13.78%), Lorestan, a province of western Iran (15.4%), and Kermanshah (8.02%) in the western part of the country [12, 14–17]. Moreover, the seroprevalence rate of CE reported in this study is lower than those reported from the hot regions of Iran, including Isfahan (1.1%), Qom (1.6%), Markazi (3.46%), and Kashan (3.05%) in Central Iran and cold area including East Azerbaijan (1.28%), Hamedan (0.4%), and North Khorasan (3.96%) [18–25].

Rural life is always considered an important risk factor in obtaining the hydatid cyst. The type of livelihood of people, which is mainly animal husbandry and agriculture, keeping dogs, and low level of health and access to health services, contributes to the higher prevalence of the disease in rural areas [26, 27].

Findings of the current study revealed higher seropositivity of hydatid cyst in women (10.51%) than in men (6.94%). In most areas of Iran especially in rural areas, women are more likely to be infected with hydatid cyst than men due to their risky behaviors such as close contact with dogs, cleaning vegetables, contact with soil, animal husbandry, and working on farms [28, 29].

Kavar County, where the present study was conducted, has a suitable climate for agriculture and animal husbandry. People in this area have not yet given up rural life, and many people have close contact with livestock and dogs, which justifies the high prevalence of hydatid cyst in the area.

In the previous studies, the rate of *Echinococcus* infection in the final host (mainly dogs) in the Fars province in Iran, where the current study has been undertaken, has been reported to be relatively high. In Mehrabani et al. study, the infection rate of dogs with *Echinococcus* adult worms in 105 dogs studied in Shiraz, the capital of Fars province, was reported to be as high as 36.19% [30]. A recent multivariate model predicting study on human CE in Fars province reported that the occurrence of CE in Fars province is affected mainly by an urban setting and the densities of cattle and dogs [31].

Studies on the *Echinococcus* genotypes in dogs in Iran have documented that dog in different regions of the country is mainly infected with G1-G3 genotypes which is the dominant genotype in humans in Iran [32].

In the present study, the subjects were divided into three age groups: 35-45, 46-55, and 56-70 years. The highest seropositivity (11.8%) was observed in the 35-45 age group. Also, multivariate logistic regression showed that the age group of 35-45 years old was 2.23 times more likely to be seropositive for CE than other age groups. In several serosurveys conducted in Iran, the age groups of 20 to 40 years old had the highest seroprevalence rate of hydatid cyst which is somewhat consistent with the findings of our study [12, 16, 25, 28]. In studies conducted in Isfahan in Central, Ardabil in northwest, and Hamedan in the western areas of Iran, the highest rate of seropositivity to hydatid cyst was seen in people over 60 years of age, which again indicates the high prevalence of infection at older ages [18, 33, 34]. In a study by Sarkari et al. on seroprevalence of hydatid cyst in children in a rural area of Kazerun, southern Iran, a low prevalence of infection in this group was reported. This is related to the nature of hydatid cyst, which has a slow growth in humans, which results in the appearance of the disease in older people, as well as the high seroprevalence of hydatid cyst in older ages [35, 36]. It is worth mentioning that, with age, the chances of contact with disease-related factors increase, and as a result, the prevalence of hydatid cyst increases at an older age.

We also found a statistically significant association between a few underlying diseases and seropositivity to hydatid cyst. In some studies, cases of arterial hypertension due to pressure from hydatid cysts have been reported [37, 38]. However, in the present study, the presence of cysts in the liver of seropositive individuals has not been determined; so, arterial hypertension in these individuals cannot be easily attributed to hydatid cysts. Fatty liver was another disease that was statistically associated with seropositivity to hydatid cyst. This may be an accidental finding, as there is no evidence to support any link between fatty liver and hydatid cyst [39].

It has been documented that the native antigen B of *E. granulosus* is the most appropriate antigen for serodiagnosis of CE [40]. In recent years, the use of recombinant antigen B has shown advantages over the native antigen [7, 41, 42] In the present study, we used the recombinant B8/1 subunit of antigen B for the detection of anti-hydatid cyst antibodies in the sera of the studied population. This antigen showed 92% sensitivity and 93% specificity in diagnosis CE in our previous study [7]. This antigen has also been used in our previous study to investigate the seroprevalence of hydatid cyst in North Khorasan province, Northeast Iran [25].

One of the shortcomings of this study is the limited age range of the subjects, which is due to the population under study in the Persian cohort, which does not include children.

## 5. Conclusion

The findings of the current study determined the serostatus of hydatid cyst in a relatively large population in Kavar County in Fars province, southern Iran. The findings indicated a relatively high rate of seropositivity to hydatid cysts and highlighted the importance and related risk factors of the disease, in a CE-endemic area in Iran. Considering the findings of the study, educating people and implementing preventive measures for the control of the disease in the region seem necessary.

## Figures and Tables

**Figure 1:** Map of the study area, Kavar County in Fars province, southern Iran.

**Table 1:** Demographic features and their relative with hydatid cyst in 1500 subjects in Kavar County, Fars province, southern Iran.

Characteristics	Frequency	Percent (%)	Seropositive for antihydatid cyst antibodies		*p* value
			No	Percent	
Age group/year					0.01
35-45	485	32.3	57	11.8	
46-55	617	41.1	48	7.8	
56-70	398	26.5	26	6.5	
Total	1500	100	131	8.73	
Sex					0.02
Male	749	49.9	52	6.94	
Female	751	50.1	79	10.51	
Education					0.25
Illiterate	479	31.9	31	6.5	
Elementary	493	32.9	49	9.4	
Middle school	229	15.3	21	9.2	
High school	166	11.1	20	12	
Associate degree	39	2.3	1	2.6	
Bachelor's degree	74	4.9	8	10.8	
Master degree	17	1.1	1	5.9	
PhD	3	0.2	0	0	
Occupation					0.008
Housekeeper	700	46.7	73	10.4	
Unemployment	230	15.4	27	11.7	
Driver	139	9.3	6	4.3	
Employee	89	5.9	10	11.2	
Seller	124	8.3	5	4	
Manual worker	99	6.6	5	5.1	
Farmer	104	6.9	3	2.9	
Rancher	15	1	2	13.3	
Animal contact level					0.84
Discontinuous	525	35	47	8.9	
Continuous	975	65	84	8.6	

## Data Availability

Data used to support the findings of this study are included in the article.
